# Development and Validation of Prediction Equation of “Athens Authentic Marathon” Men’s Race Speed

**DOI:** 10.3389/fphys.2021.682359

**Published:** 2021-07-01

**Authors:** Pantelis T. Nikolaidis, Thomas Rosemann, Beat Knechtle

**Affiliations:** ^1^School of Health and Caring Sciences, University of West Attica, Egaleo, Greece; ^2^Exercise Physiology Laboratory, Nikaia, Greece; ^3^Institute of Primary Care, University of Zurich, Zurich, Switzerland; ^4^Medbase St. Gallen am Vadianplatz, St. Gallen, Switzerland

**Keywords:** aerobic capacity, anthropometry, body composition, distance running, male, physical activity, physiology, training

## Abstract

**Aim:**

Despite the increasing popularity of outdoor endurance running races of different distances, little information exists about the role of training and physiological characteristics of recreational runners. The aim of the present study was (a) to examine the role of training and physiological characteristics on the performance of recreational marathon runners and (b) to develop a prediction equation of men’s race time in the “Athens Authentic Marathon.”

**Methods:**

Recreational male marathon runners (*n* = 130, age 44.1 ± 8.6 years)—who finished the “Athens Authentic Marathon” 2017—performed a series of anthropometry and physical fitness tests including body mass index (BMI), body fat percentage (BF), maximal oxygen uptake (VO_2_max), anaerobic power, squat, and countermovement jump. The variation of these characteristics was examined by quintiles (i.e., five groups consisting of 26 participants in each) of the race speed. An experimental group (EXP, *n* = 65) was used to develop a prediction equation of the race time, which was verified in a control group (CON, *n* = 65).

**Results:**

In the overall sample, a one-way ANOVA showed a main effect of quintiles on race speed on weekly training days and distance, age, body weight, BMI, BF, and VO_2_max (*p* ≤ 0.003, η^2^ ≥ 0.121), where the faster groups outscored the slower groups. Running speed during the race correlated moderately with age (*r* = −0.36, *p* < 0.001) and largely with the number of weekly training days (*r* = 0.52, *p* < 0.001) and weekly running distance (*r* = 0.58, *p* < 0.001), but not with the number of previously finished marathons (*r* = 0.08, *p* = 0.369). With regard to physiological characteristics, running speed correlated largely with body mass (*r* = −0.52, *p* < 0.001), BMI (*r* = −0.60, *p* < 0.001), BF (*r* = −0.65, *p* < 0.001), VO_2_max (*r* = 0.67, *p* < 0.001), moderately with isometric muscle strength (*r* = 0.42, *p* < 0.001), and small with anaerobic muscle power (*r* = 0.20, *p* = 0.021). In EXP, race speed could be predicted (*R*^2^ = 0.61, standard error of the estimate = 1.19) using the formula “8.804 + 0.111 × VO_2_max + 0.029 × weekly training distance in km −0.218 × BMI.” Applying this equation in CON, no bias was observed (difference between observed and predicted value 0.12 ± 1.09 km/h, 95% confidence intervals −0.15, 0.40, *p* = 0.122).

**Conclusion:**

These findings highlighted the role of aerobic capacity, training, and body mass status for the performance of recreational male runners in a marathon race. The findings would be of great practical importance for coaches and trainers to predict the average marathon race time in a specific group of runners.

## Introduction

The number of marathon races and runners has increased largely during the last decades (Knechtle et al., 2020; Vitti et al., 2020). For instance, the number of finishers in the New York City Marathon doubled from the 1980s to the 2010s (Vitti et al., 2020). This implied that many runners competed in a marathon race for their first time or had a small sport experience, and consequently, the need to aid such runners has been documented (Keogh et al., 2020; Malchrowicz-Mośko et al., 2020). An important question in recreational marathon runners has been the selection of a realistic goal, i.e., race pace that would allow a successful finish. In this context, researchers have attempted to develop prediction equations of marathon race speed or marathon race time (Alvero-Cruz et al., 2020; Doherty et al., 2020). For instance, Alvero-Cruz et al. (2020) reviewed 21 studies on predictors of marathon race performance from 1975 to 2020 and highlighted the role of physiology and training.

The variables included in such prediction equations might be roughly classified into three distinct groups: anthropometry, physiology and training (Foster, 1983; Tanda, 2011). Body mass index (BMI; Doherty et al., 2020), body fat percentage (BF; Salinero et al., 2017), skinfold thickness (Arrese and Ostáriz, 2006), and somatotype (Bale et al., 1985) have been used among anthropometric-related variables, where high scores in BMI or fat indices were associated with a slower race speed. The physiological variables included maximal oxygen uptake (VO_2_max; Hagan et al., 1981), submaximal VO_2_, anaerobic threshold (Esteve-Lanao et al., 2021), and submaximal blood lactate (Noakes et al., 1990) with race speed being related with higher VO_2_max and anaerobic threshold, and lower submaximal VO_2_ and blood lactate. With regard to training variables, the number of finished marathons (Doherty et al., 2020), the weekly running distance, the average training running speed (Tanda, 2011), and the duration of a training unit (Takeshima and Tanaka, 1995) have been used to predict performance in a marathon.

Although the abovementioned studies improved our understanding of performance correlates in marathon races and developed prediction equations (Alvero-Cruz et al., 2020; Doherty et al., 2020), there was a clear gap in the existing literature concerning the validation of such equations in other samples than those being developed. Moreover, a recent review of relevant prediction equations highlighted that few studies examined both anthropometric, physiological, and training variables, whereas most of previous research focused on one of these three groups of variables (Alvero-Cruz et al., 2020).

To enhance our knowledge in this area, research should be conducted not only to develop but also to validate a prediction equation. Valid equations would be a practical tool for coaches and trainers to set the target race pace for their runners. Therefore, the aim of the present study was to (a) profile anthropometric, physiological, and training characteristics of men recreational marathon runners by performance level and (b) develop and validate a prediction equation of race speed in the “Athens Authentic Marathon.” It was hypothesized that runners with a faster running speed would present better scores in the characteristics associated with performance (e.g., VO_2_max, body composition, and training) than their slower counterparts (Foster, 1983; Tanda, 2011). It was also assumed that these characteristics could be used to predict race speed in the particular marathon race.

## Materials and Methods

### Participants and Study Design

The study design was cross-sectional and included three steps: (i) comparison among performance groups based on race time on the same marathon competition; (ii) development of a prediction equation of race speed on an experimental group (EXP); and (iii) validation of this prediction equation of race speed in a control group (CON).

Participants were recreational male marathon runners (*n* = 130) who finished the “Athens Authentic Marathon” in 2017 (Table 1). They had a sport history of 6.8 ± 5.8 years of running training, number of finished marathons 5.7 ± 6.4 (best time 4:01 ± 0:45 h:min), and number of finished half-marathons 12.7 ± 16.7 (best time 1:45 ± 0:17 h:min).

**TABLE 1:** Training, anthropometric, and physiological characteristics in the total sample of participants (*n* = 130) and by quintiles of race speed.

	Total (*n* = 130)	Slow (*n* = 26)	Below average (*n* = 26)	Average (*n* = 26)	Above average (*n* = 26)	Fast (*n* = 26)	*p*	η ^2^
Race speed (km⋅h^–1^)	10.29 ± 1.87	7.62 ± 0.83^#^	9.30 ± 0.47^#^	10.50 ± 0.21^#^	11.20 ± 0.24^#^	12.84 ± 1.00^#^	< 0.001	0.889
Finished races (*n*)	5.7 ± 6.4	4.1 ± 5.9	6.1 ± 9.1	5.2 ± 5.2	7.2 ± 6.5	5.7 ± 4.1	0.526	0.025
Training days (n⋅wk^–1^)	4.4 ± 1.2	3.6 ± 1.3^AF^	3.9 ± 0.9^F^	4.1 ± 1.0^F^	4.6 ± 1.0*S*^F^	5.6 ± 1.1^#^	< 0.001	0.299
Training distance (km⋅wk^–1^)	53.2 ± 21.0	36.5 ± 13.9^AF^	48.7 ± 13.5^F^	50.3 ± 19.7^F^	57.4 ± 21.6^SF^	72.1 ± 18.0^#^	< 0.001	0.313
Age (years)	44.1 ± 8.6	48.1 ± 6.7^AF^	45.8 ± 9.2	45.4 ± 7.9	41.5 ± 8.8^S^	40.0 ± 8.0^S^	0.003	0.121
Body height (cm)	176 ± 6	175 ± 5	177 ± 8	177 ± 5	177 ± 5	175 ± 6	0.355	0.034
Body weight (kg)	76.9 ± 9.4	82.2 ± 11.4^AF^	80.5 ± 6.7^F^	77.4 ± 7.5^F^	75.1 ± 8.6^S^	69.3 ± 6.3^SBV^	< 0.001	0.237
BMI (kg⋅m^–2^)	24.7 ± 2.6	26.7 ± 3.1^VAF^	25.6 ± 1.5^AF^	24.7 ± 2.0^SF^	23.8 ± 2.3^SB^	22.6 ± 1.3^SBV^	< 0.001	0.302
BF (%)	17.7 ± 4.1	21.1 ± 3.0^VAF^	19.0 ± 3.0^F^	18.4 ± 3.2^SF^	16.6 ± 4.0^SF^	13.4 ± 2.6^#^	< 0.001	0.404
VO_2_max (ml⋅min^–1^⋅kg^–1^)	48.3 ± 8.0	41.1 ± 6.6^VAF^	44.4 ± 6.0^AF^	48.3 ± 6.3^SF^	51.7 ± 6.2^SB^	56.2 ± 5.3^SBV^	< 0.001	0.442
Pmax (W⋅kg^–1^)	10.4 ± 1.5	10.1 ± 1.6	10.4 ± 1.7	9.9 ± 1.3	10.4 ± 1.3	10.9 ± 1.3	0.151	0.052
SAR (cm)	17.6 ± 8.5	16.4 ± 10.0	18.3 ± 8.0	16.3 ± 7.3	20.3 ± 8.6	16.9 ± 8.1	0.374	0.033
SJ (cm)	24.3 ± 4.2	23.3 ± 3.7	24.9 ± 4.2	23.6 ± 4.6	24.7 ± 3.3	25.2 ± 5.2	0.454	0.029
CMJ (cm)	25.8 ± 4.8	24.9 ± 4.6	26.3 ± 4.5	24.5 ± 5.0	26.1 ± 3.5	27.2 ± 5.9	0.237	0.043

*Values were presented as mean ± standard deviation (SD). Capital letters as exponents next to SD denote difference at *p* < 0.05 from slow (S), below average (B), average (V), above average (A), and fast group (F), and symbol ^#^ shows statistical difference from all other groups. BMI, body mass index; BF, body fat percentage; VO_2_max, maximal oxygen uptake; Pmax, maximal anaerobic power; SAR, sit-and-reach test; SJ, squat jump; and CMJ, countermovement jump.*

All procedures were in agreement with the guidelines of the Declaration of Helsinki and approved by the local Institutional Review Board (EPL 2017/3). All participants provided written informed consent prior to the exercise testing session. In this project, participants were recruited using public calls through social media and local running clubs of Athens about 6 months prior to the race of 2017. Having finished a marathon race in the past and the intention to participate in the “Athens Authentic Marathon” 2017 were prerequisites for inclusion in this study. Considering the relatively small number of women finishers in this race (men-to-women ratio ∼4, https://www.athensauthenticmarathon.gr/site/index.php/el/results-gr/496-results-2017-marathon-gr), only men were included in the present analysis.

It was acknowledged that groups of specific race time ranges (e.g., 3:00–3:30 h:min versus 3:30–4:00 h:min) could be also used as a methodological approach instead of quintiles of race speed. Nevertheless, quintiles of race speed were qualified as better descriptors of performance independently from marathon race, since performance might vary among marathon races. A methodological approach to consider performance groups of marathon runners based on relative performance (e.g., quartiles) instead of absolute performance (e.g., race time) has been used previously (Hopkins and Hewson, 2001; Bobbert et al., 2012; Brown and Scurr, 2016; Stones, 2019). Thus, participants in the present study were grouped according to quintiles of race speed into slow (5.95–8.47 km/h), below average (8.48–10.13 km/h), average (10.14–10.81 km/h), above average (10.82–11.56 km/h), and fast group (11.57–15.00 km/h). In addition, participants were randomly classified into two equal-size groups matched for performance, an experimental (EXP, *n* = 65) group and a control (CON, *n* = 65) group. EXP provided data to develop an equation predicting race speed, and thereafter, predicted race speed was calculated for CON.

### Equipment and Protocols

All participants performed a series of anthropometry and physical fitness tests including BMI, BF, VO_2_max, sit-and-reach test (SAR), isometric muscle strength, anaerobic power (force–velocity test), squat jump (SJ), and countermovement jump (CMJ) about 1 month prior to the “Athens Authentic Marathon.” Details for equipment and testing protocols have been described elsewhere (Nikolaidis and Knechtle, 2018).

In SAR, SJ, and CMJ, two trials were performed and the best one was recorded for further analyses; the intraclass correlation coefficient (ICC) of these tests was 0.99. Body height was evaluated using a stadiometer (SECA, Leicester, United Kingdom) and body weight by an electronic scale (HD-351; Tanita, Arlington Heights, IL, United States), and these variables were used to calculate BMI. Skinfold thickness of 10 sites (Harpenden caliper, Baty International, West Sussex, United Kingdom) was measured (Eston and Reilly, 2001). VO_2_max was measured in a graded exercise test (GXT) with an initial speed set at 8 km/h, an inclination 1%, and an increase of speed by 1 km/h every minute. Lactate concentration was evaluated 5 min after finishing GXT (Accutrend, Roche, Germany). During GXT, HR was monitored by Team2 Pro (Polar Electro Oy, Kempele, Finland), and VO_2_ by a gas analyzer (Fitmate PRO, COSMED, Rome, Italy).

Low-back and hamstring flexibility was evaluated by SAR (Mayorga-Vega et al., 2014) on a box providing a 15-cm advantage (ICC 0.98). Isometric muscle strength was evaluated as the sum of four tests (right and left handgrip test, back test, and back-and-leg test) using dynamometers (Takei, Tokyo, Japan) relative to body weight values (ICC 0.95; Heyward, 2010). SJ and CMJ (Aragón, 2000) were tested in the Optojump photoelectronic system (Microgate Engineering, Bolzano, Italy; SJ, ICC 0.91; CMJ, ICC 0.95). Muscle power (Pmax) was evaluated using the *F-v* test on a leg cycle ergometer (Ergomedics 874E, Monark, Sweden; Vandewalle et al., 1985). It should be noted that, despite the limited evidence of the relevance of flexibility, muscle strength, and power with performance (Piacentini et al., 2013; Del Coso et al., 2019), their evaluation might provide a more complete physiological profile of marathon runners.

### Statistical and Data Analysis

GraphPad Prism v. 7.0 (GraphPad Software, San Diego, CA, United States) and IBM SPSS v. 23.0 (SPSS, Chicago, IL, United States) conducted the statistical analyses. Statistical significance was set at alpha = 0.05. The Kolmogorov–Smirnov test and visual inspection of Q–Q plots tested the normality of the data. A one-way analysis of variance (ANOVA) examined differences in anthropometric, physiological, and training characteristics among performance groups. The magnitude of differences was evaluated using eta squared. The Pearson moment correlation coefficient (r) evaluated the relationship of race speed with the abovementioned characteristics. An independent *t*-test examined differences in training, anthropometric, and physiological characteristics between EXP and CON. The magnitude of this comparison was evaluated using Cohen’s d. A stepwise linear regression was used to develop a prediction equation of race speed in EXP. Age and training (number of finished marathons, training sessions, and running distance per week) and anthropometric (body weight, body height, BMI, BF, FFM, circumferences, and WHR) and physiological characteristics (VO_2_max, HRmax, lactate, Pmax, isometric muscle strength, SJ, CMJ, and SAR) were considered as potential predictor variables. Stepping method criteria consisted of using probability *F* ≤ 0.05 for entry and *F* ≥ 0.10 for removal. The agreement between actual and predicted race speed was examined in the CON Bland–Altman plot.

## Results

A one-way ANOVA showed a main effect of quintiles of race speed on weekly training days and distance, age, body weight, BMI, BF, and VO_2_max (*p* ≤ 0.003, η^2^ ≥ 0.121), where the faster groups outscored the lower groups (Table 1). The magnitude of this effect was large except in the case of age, where it was moderate. It should be highlighted that weekly training days and distance and BF were variables were fast, differing from the above average runners.

Running speed during the race correlated moderately with age (*r* = −0.36, *p* < 0.001) and largely with the number of weekly training days (*r* = 0.52, *p* < 0.001) and weekly running distance (*r* = 0.58, *p* < 0.001), but not with the number of previously finished marathons (*r* = 0.08, *p* = 0.369). With regard to physiological characteristics, running speed correlated largely with body mass (*r* = −0.52, *p* < 0.001), BMI (*r* = −0.60, *p* < 0.001), BF (*r* = −0.65, *p* < 0.001), and VO_2_max (*r* = 0.67, *p* < 0.001), moderately with isometric muscle strength (*r* = 0.42, *p* < 0.001), and little with anaerobic muscle power (*r* = 0.20, *p* = 0.021), but not with SAR (*r* = 0.06, *p* = 0.491), SJ (*r* = 0.13, *p* = 0.158), and CMJ (*r* = 0.13, *p* = 0.131; Figure 1).

**FIGURE 1:** Relationship of race speed with weekly running distance, maximal oxygen uptake, and body mass index in the total sample of male marathon runners (*n* = 130). VO_2_max, maximal oxygen uptake; BMI, body mass index. The shaded band around the regression line denotes the 95% confidence interval on this line.

Compared to CON, EXP did not differ in age (mean difference −1.4 years; 95% confidence intervals, CI, −4.4, 1.6), body height (−0.3 cm; 95% CI −2.3, 1.8), body weight (−0.7 kg; 95% CI −3.9, 2.6), BMI (−0.1 kg⋅m^–2^; 95% CI −1.0, 0.8), BF (1.0%; 95% CI −0.5, 2.4), VO_2_max (−0.4 ml⋅min^–1^⋅kg^–1^; 95% CI −3.3, 2.4), Pmax (0.1 W⋅kg^–1^; 95% CI −0.4, 0.7), SAR (−1.5 cm; 95% CI −4.4, 1.4), SJ (0 cm, 95% CI −1.5, 1.4), and CMJ (−0.1 cm; 95% CI −1.8, 1.5). In addition, the two groups did not differ in race speed (−0.1 km/h; 95% CI −0.7, 0.6), number of finished marathon races (−0.6; 95% CI −2.8, 1.6), weekly training days (−0.3; 95% CI −0.7, 0.2), and distance (−5.9 km; 95% CI −13.2, 1.5; Table 2).

**TABLE 2:** Training, anthropometric, and physiological characteristics in the experimental (*n* = 65) and control group (*n* = 65).

	EXP (*n* = 65)	CON (*n* = 65)	*p*	*d*
Race speed (km⋅h^–1^)	10.26 ± 1.87	10.33 ± 1.88	0.834	0.04
Finished races (*n*)	5.4 ± 5.6	6.0 ± 7.1	0.598	0.09
Training days (n⋅wk^–1^)	4.2 ± 1.3	4.5 ± 1.2	0.215	0.24
Training distance (km⋅wk^–1^)	50.3 ± 18.7	56.2 ± 22.9	0.117	0.28
Age (years)	43.4 ± 8.3	44.9 ± 8.8	0.347	0.18
Body height (cm)	176 ± 6	177 ± 6	0.804	0.17
Body weight (kg)	76.6 ± 9.3	77.2 ± 9.5	0.691	0.06
BMI (kg⋅m^–2^)	24.6 ± 2.6	24.7 ± 2.5	0.769	0.04
BF (%)	18.2 ± 3.7	17.2 ± 4.4	0.186	0.25
VO_2_max (ml⋅min^–1^⋅kg^–1^)	48.1 ± 7.1	48.6 ± 8.9	0.752	0.06
Pmax (W⋅kg^–1^)	10.4 ± 1.4	10.3 ± 1.6	0.574	0.07
SAR (cm)	16.9 ± 8.0	18.4 ± 8.9	0.314	0.18
SJ (cm)	24.3 ± 4.0	24.4 ± 4.5	0.950	0.02
CMJ (cm)	25.7 ± 4.6	25.9 ± 5.0	0.884	0.04

*Values were presented as mean ± standard deviation (SD). BMI, body mass index; BF, body fat percentage; VO_2_max, maximal oxygen uptake; Pmax, maximal anaerobic power; SAR, sit-and-reach test; SJ, squat jump; and CMJ, countermovement jump.*

Race speed in EXP could be predicted (*R*^2^ = 0.61, standard error of the estimate = 1.19) using the formula “8.804 + 0.111 × VO_2_max + 0.029 × weekly training distance in km − 0.218 × BMI” (Table 3). Applying this equation in CON, no bias was observed (difference between observed and predicted value 0.12 ± 1.09 km/h, 95% confidence intervals −0.15, 0.40, *p* = 0.122; Figure 2).

**TABLE 3:** Model summary of stepwise regression in the experimental group (*n* = 65).

Model	Predictors	*R*	*R*^2^	SEE
1	VO_2_max	0.65	0.41	1.44
2	VO_2_max, weekly distance	0.73	0.52	1.30
3	VO_2_max, weekly distance, BMI	0.78	0.59	1.20

*VO_2_max, maximal oxygen uptake; BMI, body mass index; *R*, correlation coefficient; *R*^2^, coefficient of determination; and SEE, standard error of the estimate.*

**FIGURE 2:** Bland–Altman plot describing the agreement between actual and predicted race speed in the Athens marathon race. The *Y*-axis shows the difference between actual and predicted score, whereas the *X*-axis represents the average of actual and predicted score.

## Discussion

The main findings of the present study were that (a) the faster groups outscored the lower groups in weekly training days and distance, age, body weight, BMI, BF, and VO_2_max; (b) race speed correlated largely with the number of weekly training days, weekly running distance, body mass, BMI, BF, and VO_2_max, moderately with age, and small with the anaerobic muscle power; (c) race speed in EXP could be predicted by VO_2_max, weekly training distance, and BMI, confirming our research hypothesis; and (d) applying the developed equation in CON, no bias was observed. Also, it should be underlined that CON and EXP did not differ in any anthropometric, physiological, or training variable.

The best predictor of race speed was VO_2_max, explaining a large portion of variance (∼40%). This finding was in agreement with previous research including VO_2_max in prediction equations of race speed or time (Foster, 1983). Moreover, it was in line with a comparative study of recreational marathon runners of different performance levels showing that the faster runners had higher VO_2_max than the slower ones (Gordon et al., 2017). The role of VO_2_max for marathon performance highlighted the need of a well-developed cardiorespiratory (to transfer O_2_ to skeletal muscles) and muscular system (to metabolize O_2_).

The weekly training distance was the second entered variable in the regression model, highlighting the importance of training for performance. This observation came to terms with previous studies on long-distance runners’ training characteristics (Slovic, 1977; Foster, 1983). For instance, marathon race time was related with the longest training distance and running pace during 8 weeks prior to a race (Foster, 1983). Moreover, Slovic (1977); Hagan et al. (1981, 1987), and Tanda and Knechtle (2013) reported that marathon race time was associated with the overall training distance in addition to the running pace and the longest distance completed prior to race. An explanation for this finding was the favorable physiological adaptations to long-term endurance exercise with regard to parameters related to endurance performance such as VO_2_max.

The third entered variable in the regression model was BMI. This finding was in agreement with previous research showing that an increased BMI was related to slower race time in marathon (Hagan et al., 1987; Doherty et al., 2020), half-marathon (Campbell, 1985; Rüst et al., 2011; Friedrich et al., 2014; Gómez-Molina et al., 2017), and 10 km (Berg et al., 1998). These findings highlighted the negative role of an increased BMI on long-distance running performance, since an excess weight should be carried throughout the distance; the excess weight quantitatively might be more important than the quality of this excess weight (i.e., fat or fat-free mass). In contrast to BMI, BF was not a predictor of race speed in the present study, which was in line with studies observing that a measure of BF (e.g., skinfolds, circumferences) played a less important role than BMI for performance (Friedrich et al., 2014; Rüst et al., 2011).

Although age correlated moderately with race time and fast participants were ∼8 years younger than slow participants, age was not a predictor of race time according to the statistical model used in the present study. Considering the 21 previous studies on race time predictors reviewed by Alvero-Cruz et al. (2020), age was included in a prediction equation only in two studies (Hagan et al., 1981; Keogh et al., 2020). An explanation for why age was not a predictor of race time in our study—similarly to the majority of previous studies—might be the relationship of age with predictors of race time such as VO_2_max (Rogers et al., 1990) and BMI (Wang et al., 2007), where an older age was related to a lower VO_2_max and a larger BMI. It should be highlighted that the age of participants was similar to the age previously reported for men marathon runners in Switzerland (Knechtle et al., 2016b), where elite runners (East Africans) were younger by 13.5 years than recreational runners (Knechtle et al., 2016a). It was assumed that the relationship of age with race time might vary by performance level, e.g., a lower decline of performance with aging might be observed in recreational than in elite runners (Zavorsky et al., 2017), which might explain the magnitude of this relationship in the present study. Moreover, the relationship of race time with measures of muscle strength and power such as SJ, CMJ, anaerobic power, and isometric muscle strength ranged from trivial to moderate, indicating the small affinity of these measures with a sport relying mostly on aerobic capacity (Tam et al., 2012). This observation was in agreement with research showing that long-distance runners had the lowest SJ compared to combat sports, power track and field, racket sports, and team sports (Valenzuela et al., 2020).

With regard to the findings of the validation study, no difference was observed in race speed between actual and predicted scores in CON. This finding was of great practical application suggesting the further use of this equation in other samples of male recreational runners to predict their speed in marathon races with similar characteristics with “Athens Authentic Marathon.” It should be highlighted that the value of this equation was to predict the mean score of a group of runners and not individual scores. An explanation of this discrepancy among individual scores might be that ∼40% of the observed variance in race speed was attributed to other parameters than those (VO_2_max, training distance, and BMI) included in the prediction equation. The “other” parameters referred to aspects such as psychological characteristics, technological aids (e.g., shoes), nutritional strategies, and potential use of drugs (Joyner et al., 2020).

A limitation of the present study was the included variables in the regression analysis to identify predictors of race time. It should be clarified that the predictors of race time derived from a stepwise regression analysis were considered in the light of the included variables. It was acknowledged that the predictors could differ in the case that other variables (e.g., nutrition, psychology, biomechanics, and physical readiness) were included in the model (Alvero-Cruz et al., 2020). Taking into account differences among marathon races [the “Athens Authentic Marathon” had a minimum elevation 7 m and a maximum elevation 244 m (Nikolaidis and Knechtle, 2018) compared to flat marathons such as the six World Marathon Majors (Díaz et al., 2019)] and runners of various performance levels (the mean race time was 4:06 h:min in our sample), caution would be needed to generalize the findings of the present study in other races and samples of marathon runners (Oficial-Casado et al., 2020).

Furthermore, it was acknowledged that a larger sample size would allow including more variables as candidate predictors of race performance. It should be noted that Alvero-Cruz et al. (2020) reported men’s sample sizes of 21 studies on predictors of marathon race performance ranging from 8 (Esteve-Lanao et al., 2021) to 166 (Roecker et al., 1998). In this context, our sample size might be considered one of the largest ever used to predict marathon race performance. In addition, a potential increase of the sample size would prolong the period between testing and race and, consequently, decrease the predicting value of VO_2_max, BMI, and weekly running distance (Esteve-Lanao et al., 2021). The results would have large practical applications for coaches and trainers working with recreational marathon runners to set pace during the race. That is, the administration of a GXT to assess VO_2_max, evaluation of weight status, and recording of weekly running distance within a short period (Esteve-Lanao et al., 2021) prior to a marathon race might help runners for an optimal race pace. Considering the findings on the role of BMI for performance, recreational marathon runners should be advised to focus mostly on their weight control rather than BF.

## Conclusion

The results of the present study highlighted the role of aerobic capacity, training, and body mass status for the performance of recreational male runners in a marathon race. These findings would aid professionals working with men marathon runners predicting the average marathon race time in a group of runners. Future research should use a multicenter study design—where several laboratories could be recruited to evaluate larger samples of marathon runners with reference to the same marathon race—in order to include more variables as candidate predictors of race time. In this way, it would be possible to predict not only average scores for a group of runners but also individual race times.

## Data Availability Statement

The raw data supporting the conclusions of this article will be made available by the authors, without undue reservation.

## Ethics Statement

The studies involving human participants were reviewed and approved by All procedures were in agreement with the guidelines of the Declaration of Helsinki, and approved by the local Institutional Review Board (EPL 2017/3). All participants provided written informed consent prior to exercise testing session.

## Author Contributions

PN collected the data and drafted the manuscript. TR and BK helped in drafting the manuscript. All authors contributed to the article and approved the submitted version.

## Conflict of Interest

The authors declare that the research was conducted in the absence of any commercial or financial relationships that could be construed as a potential conflict of interest.
